The article "Using Machine Learning to Predict the Requirement for Revascularization in Patients with Chest Pain in the Emergency Department" was published in 2022. Journal: J Healthc Eng.

# Using Machine Learning to Predict the Requirement for Revascularization in Patients with Chest Pain in the Emergency Department

**DOI:** 10.1155/2022/1795588

**Published:** 2022-04-14

**Authors:** ZhiChang Zheng, Ruifeng Guo, Nian Wang, Bo Jiang, Chun Peng Ma, Hui Ai, Xiao Wang, ShaoPing NIE

**Affiliations:** ^1^Center for Coronary Artery Disease, Division of Cardiology, Beijing Anzhen Hospital, Capital Medical University, Anzhen Road Chaoyang District, Beijing 100029, China; ^2^Department of Cardiology, Beijing Bo'ai Hospital, China Rehabilitation Research Center, Capital Medical University, No. 10 Jiaomen North Road Fengtai District, Beijing 100068, China; ^3^State Key Laboratory of Software Development Environment, School of Computer Science and Engineering, Beihang University, Beijing 100191, China; ^4^Department of Cardiology, the First Hospital of Qinhuangdao, Hebei Medical University, Qinhuangdao 066099, Hebei, China

## Abstract

**Objective:**

The study aimed to use machine learning algorithms to predict the need for revascularization in patients presenting with chest pain in the emergency department.

**Methods:**

We obtained data from 581 patients with chest pain, 264 who underwent revascularization, and the other 317 were treated with medication alone for 3 months. Using standard algorithms, linear discriminant analysis, and standard algorithms, we analyzed 41 features relevant to coronary artery disease (CAD).

**Results:**

We identified seven robust predictive features. The combination of these predictors gave an area under the curve (AUC) of 0.830 to predict the need for revascularization. By contrast, the GRACE score gave an AUC of 0.68.

**Conclusions:**

This machine learning-based approach predicts the need for revascularization in patients with chest pain.

## 1. Background

Chest pain is among the most common complaints of patients in the emergency or cardiology outpatient department. Because of the severity of the consequences of many etiologies of chest pain, rapid evaluation is critical. Many patients undergo coronary computed tomography angiography or coronary angiography (CAG) because chest pain may signal coronary artery disease (CAD).

Routine use of risk scores might improve decision-making. The Global Registry of Acute Coronary Events (GRACE) score evaluates the outcomes in patients with CAD, particularly those with acute coronary syndrome [1]. Current guidelines call for aggressive management, including revascularization in at-risk patients [2]. For patients with chest pain, revascularization is one of the effective ways to lower the rates of myocardial infarction or death. Importantly, for some patients with serious chest pain, the coronary arteries might become more severely blocked and require a revascularization procedure as soon as possible. Nevertheless, there are data suggesting that patients at low risk of developing ischemic complications are treated overly aggressively, generating the so-called “treatment-risk paradox” [3–5]. For this reason, there is a need for prediction models in addition to the GRACE risk score [6].

In recent years, we have developed software applications such as data engineering, data architecture, and machine learning (ML). The latter are algorithms that identify patterns embedded in large datasets containing large numbers of variables. Machine learning for detection and diagnosis of disease is a hot research area in recent years. Machine learning offers a principled approach for developing automatic, sophisticated, and objective algorithms for analysis of high-dimensional and substantial biomedical data. ML enables the generation of predictive models and disease classification models [7]. The ML system could tell us the possible diseases and risks based on given symptoms as the input. These technologies already showed great success in electrocardiography [8] and image analysis [9].

In the present study, we used an ML algorithm to generate a predictive model to identify patients with chest pain at high risk for cardiovascular events. Such patients would benefit from immediate revascularization either in the cardiology outpatient or emergency department.

## 2. Methods

### 2.1. Datasets

We used a derivation cohort of 585 adult patients (≥18 years) with chest pain who underwent invasive CAG to develop the ML models. These patients were admitted to the Emergency Department of Anzhen Hospital, Beijing, China, between 1 May 2017 and 31 January 2018. CAG was performed if aortic dissection and pulmonary embolism were tentatively excluded and if the patient exhibited symptoms that were consistent with CAD or if tests results suggested cardiac ischemia. Excluding four patients with missing critical data, a total of 581 patients were finally enrolled. Two interventional cardiologists performed coronary angiographies. All patients provided informed written consent. The institutional review board approved this study.

To assess the performance of the models, we used an external validation cohort including 172 adult patients admitted with CAD from the China Rehabilitation Research Center, Beijing, China, who underwent CAG to assess coronary artery.

### 2.2. Outcomes

We used the classification ML model to predict the occurrence of revascularization or medication alone. Patients undergoing revascularization were defined as having significant coronary artery stenosis; these patients underwent percutaneous coronary intervention or coronary bypass grafting. Patients with no evidence of significant stenotic lesion were treated with medication alone for 3 months. A total of 264 patients underwent revascularization treatment, and the remaining 317 patients received only drug therapy. We trained the classification model with data from existing patients, and then, we used the trained model to make predictions based on the data of external patients.

### 2.3. ML Method

The ML was run on Python 3.7.3 (www.python.org). The entire process of ML prediction included data preprocessing, classification using support-vector machines as the classifier, and verification using a 10-fold cross-validation method. Data preprocessing included discretization of data classified by continuous values according to the range, feature selection by the chi-square test, and feature dimension reduction using linear discriminant analysis. The ML method used the scikit-learn open-source library.

### 2.4. Feature Selection and Data Preprocessing

The structured dataset included 41 variables (Table 1). In the training set, there were 581 instances, among which 264 instances were labeled class 1 (revascularization treatment) and 317 instances were labeled as class 0 (medication treatment). In the validation dataset, there are 172 instances with 41 attributes. Of these, 39 instances were class 1 (revascularization treatment) and 133 instances were class 0 (medication treatment).

By calculating the chi-squared value of each attribute and the classification result of the training dataset, the chi-squared value of each attribute was sorted (Figure 1).

To simplify the explanation of the model from the clinical perspective, we set the upper limit of the number of selected features to 20. Of these, seven features were strongly correlated with the outcome event. The seven features selected were neutrophil-to-lymphocyte ratio, ST-segment changes, cardiac markers, lymphocyte count, lactate dehydrogenase, gender, and history of hyperlipidemia.

### 2.5. Dimensionality Reduction

After feature selection, we performed dimensionality reduction to reduce the multidimensional input data to one dimension. To be specific, we used the linear discriminant analysis feature dimension reduction method.

To perform receiver operating characteristic (ROC) curve analysis, we used the decision function of the linear support-vector classifiers to generate probabilistic outputs of the predictions; then, probabilities were used to plot the ROC curves.

### 2.6. Validation

To evaluate the accuracy of the trained classification model, we used 10-fold cross-validation. To determine whether the classifier was overfitted, we prepared a new validation dataset. The new validation dataset underwent the same data preprocessing process (i.e., data discretization, feature selection, and dimension reduction) as the training data. Finally, the preprocessed validation dataset was fed into the classification model for prediction.

## 3. Results

The area under the curve (AUC) of ML for the training set showed the best performance, with a value of 0.83; by contrast, the GRACE score AUC was 0.68 (*P* < 0.05 for the comparison). The precision value for class 0 was 0.88 in the training set and 0.86 in the validation set. The recall was also high for class 0 (medication treatment) in the validation set. The accuracy of the trained model on the training set was 75 (Figure 2). The AUC for the validation set was 0.79 (Figure 3). The classification report is given in Table 2.

## 4. Calibration

We performed model calibration to calculate the certainty of new observations in either of the established classes. The Brier score for ML was 0.212 before and 0.162 after calibration. This finding suggests a slight difference between the predicted and observed probabilities of treatment strategies and a good overall fit for the model (Figure 4).

## 5. Discussion

We used ML algorithms to predict the requirement for revascularization in patients with chest pain using basic clinical information. The AUC for the predictive value was 0.83 in the training set and 0.79 in the external validation set. These results suggest that our ML algorithm can help developing treatment strategies for individual patients with chest pain. We found that ML was 75% accurate in predicting strategies with an AUC of 0.83 in the training set. In the external data validation, ML reached 76% accuracy with an AUC of 0.79; ML had 88% precision for predicting treatment strategies, especially for medication-treated patients in the training set; and ML reached 86% precision and 81% recall for predicting medication-treated patients in the external data validation.

In the training set, ML's predictive accuracy for patients treated with medication was higher (0.88); however, the recall was lower at 0.66. For the patients with revascularization treatment, the accuracy was 0.66, the recall was 0.88, and overall accuracy was 0.83. When validated with external data, the ML's prediction model performed well for patients treated with medication, with accuracy set recalls of 0.86 and 0.81, respectively; however, the prediction for revascularization therapy was poor and performed less well than the prediction for medication therapy. The prediction of overall patient outcome, with a ROC value of 0.83 for ML, was better than the GRACE score of 0.68. We also found that, with proper calibration, the prediction of outcome events can be enhanced. Implementation of ML models in clinical settings can automate the selecting candidates who might benefit most from additional diagnostic testing while avoiding the need for time-consuming and unnecessary routine clinical steps.

Correctly identifying patients at high risk will facilitate the patients to receive appropriate treatment and improve clinical outcomes. The GRACE risk score is a validated predictor of adverse outcomes in CAD patients, and recent studies showed that the GRACE score could assess the severity of coronary artery stenosis in patients with CAD [10, 11]. Current guidelines recommend the GRACE risk score to perform risk stratification in CAD, especially for patients with acute coronary syndrome [12]. Even though the GRACE score is easy to apply, the score in isolation was associated with significant over and undertreatment, suggesting the need for more accurate assessments using a wider range of clinical variables [3, 4]. However, integrating a patient's various clinical information for risk scoring is a challenge for cardiovascular physicians. The complexity of assessment is increasing as additional clinical variables need to be considered. In general, it is challenging for cardiovascular physicians to predict risk in individual patients.

In the present study, we showed that our ML overcame these challenges, providing deep integration of comprehensive clinical data. There are some differences between our study and previous studies. Most of the latter were designed to predict the clinical outcomes after coronary artery revascularization; most relied on data from noninvasive (coronary computed tomography angiography) or invasive (coronary angiography, CAG) coronary angiographies and assistive technologies such as cardiac magnetic resonance, intravascular ultrasound, or fractional flow reserve [13, 14]. In the present study, by contrast, we used ML to predict whether patients with CAD could be treated with immediate revascularization based only on clinical data, history, and laboratory findings in the emergency department.

The ML approach is an artificial intelligence that differs from traditional prognostic methods, in which it makes no a priori assumptions regarding the cause of disease. This characteristic permits agnostic explorations of available data that may predict the risk to individuals (i.e., precise risk stratification). This approach diverges from the hypothesis-driven approach in standard prognostic risk assessment [15, 16]. We found that the precision value for class 0 (medication treatment) and the recall value for class 1 (revascularization treatment) of these two subsets were both high, especially in the training set. The recall was also high for class 0 (medication treatment) in the validation set. The high precision value of class 0 suggests that the actual class 0 instances account for a high proportion of all predicted class 0 instances, further suggesting that it is rare for the model to misjudge class 1 as class 0. The high recall value of class 1 suggests that the instances correctly identified as class 1 have a high percentage of all instances of class 1, further suggesting that the model has a high recognition accuracy for class 1. This finding was the same for the high recall value of class 0. The neutrophil-to-lymphocyte ratio showed the highest predictive weight for the outcome. The ML avoided ignoring important but unexpected predictor variables or interactions by not making the necessary prior assumptions between the cause and outcome and allowed us to identify clinically essential risks in patients with multiple marginal risk factors. Machines can quickly and seamlessly integrate new data to continuously update and optimize their algorithms, thereby continuously improving their predictive performance over time.

In general, our ML approach provided incremental gains in prognostic performance while managing 40 variables and numerous patient-specific variable-variable interactions. This process permits individualized risk assessment and circumvents several of the limitations inherent in the standard statistical approach. Our findings have considerable clinical importance. ML may help generate more accurate cardiovascular risk stratification for individual patients.

Classical statistical methods hand-pick features are based entirely on medical domain knowledge. Statistical methods are then used to calculate the importance of each feature and construct prediction models. ML methods start from the data and do not refer to traditional risk factors or weighted factors. Furthermore, they do pay attention to the interpretability of the model. It remains a challenge to fuse medical domain knowledge and ML methods to build highly interpretable predictive models. Furthermore, ML identifies risk factors different from those generated by traditional methods, allowing for more in-depth prospective studies to determine etiology and interactions. These advantages may eventually lead to new therapeutic targets [15, 17]. However, although ML methods have many application advantages, there are still some problems in its application. For example, ML methods cannot always provide rational predictions for a particular disease. ML uses extraction methods and feature representation to extract features from enormous datasets to build models without reference to known weights and risk factors. Therefore, the models are less interpretable than traditional disease prediction methods. Also, there are different ways to develop and deploy a machine learning system for specific applications, which might lead to inconsistent results.

## 6. Conclusion

We have established an ML method for predicting revascularization in patients in the emergency department with chest pain. The comparable performance with traditional models suggests the potential value of ML approaches for evaluating chest pain, which is a complex, multifactorial symptom. Although it is a method with superior advantages, the specific mechanisms of the seven clinical predictors in this ML model require further study. Longer follow-up and accumulation of multicenter data may improve ML models' sensitivity and specificity. When combined with a large and growing dataset, the ML models can be dynamically and automatically improved to achieve better performance [18].

## Figures and Tables

**Figure 1:** Feature importance plot for the machine learning model.

**Figure 2:** Area under the curve as a measure of individual model performance for the prediction in the training set.

**Figure 3:** The ROC for the validation.

**Figure 4:** Calibration slopes for the machine learning model for prediction of the likelihood of revascularization treatment.

**Table 1:** Features for analysis.

		Features
Demographic data	1	Gender
	2	Age

Clinical data at emergency or outpatient department	3	SBP
	4	DBP
	5	HR
	6	Arrhythmia
	7	ST-segment changes
	8	Killip classification

History	9	CAD
	10	MI
	11	PCI
	12	CABG
	13	Chest pain
	14	Diabetes
	15	Hypertension
	16	Stroke
	17	Hyperlipidemia
	18	PAD
	19	Smoking
	20	Drinking
	21	Family history of CHD

Laboratory data at emergency or outpatient department	22	WBC
	23	Monocyte
	24	Lymphocyte
	25	RBC
	26	HBG
	27	HCT
	28	PLT
	29	FBG
	30	Hs-CRP
	31	HCY
	32	Uric acid
	33	CRE
	34	BUN
	35	TC
	36	TG
	37	LDL-C
	38	HDL-C
	39	LDH
	40	Cardiac markers change

Calculation data	41	NLR

SBP, systolic blood pressure; DBP, diastolic blood pressure; HR, heart rate; CHD, coronary heart disease; MI, myocardial infarction; PCI, percutaneous coronary intervention; CABG, coronary artery bypass grafting; PAD, peripheral arterial disease; WBC, white blood cell; RBC, red blood cell; HGB, hemoglobin; HCT, hematocrit; PLT, platelet; FBG, fasting blood glucose; HCY, homocysteine; CRE, creatinine; BUN, blood urea nitrogen; TC, total cholesterol; TG, triglyceride; LDL, low-density lipoprotein cholesterol; HDL-C, high-density lipoprotein cholesterol; NLR, neutrophil-to-lymphocyte ratio.

**Table 2:** ML results on the training set and the validation set.

Set	Precision	Recall	F1 score	Accuracy	ROC AUC	
Training	0	0.88	0.66	0.75	0.75	0.83
	1	0.66	0.88	0.76		

Validation	0	0.86	0.81	0.84	0.76	0.79
	1	0.47	0.56	0.51		

## Data Availability

The data used to support the findings of this study are included within the article.

## Abbreviations

AUC: Area under curve
BUN: Blood urea nitrogen
CABG: Coronary artery bypass grafting
CAD: Coronary artery disease
CAG: Coronary angiography
CHD: Coronary heart disease
CRE: Creatinine
DBP: Diastolic blood pressure
FBG: Fasting blood glucose
GRACE: The Global Registry of Acute Coronary Events
HCT: Hematocrit
HCY: Homocysteine
HDL-C: High-density lipoprotein cholesterol
HGB: Hemoglobin
HR: Heart rate
LDL-C: Low-density lipoprotein cholesterol
MI: Myocardial infarction
ML: Machine learning
NLR: Neutrophil-to-lymphocyte ratio
PAD: Peripheral arterial disease
PCI: Percutaneous coronary intervention
PLT: Platelet
RBC: Red blood cell
ROC: Receiver operating characteristic curve
SBP: Systolic blood pressure
TC: Total cholesterol
TG: Triglyceride
WBC: White blood cell.
